The article "Development of Training Videos Based on Virtual Reality Side-Cut High-Simulation Simulator of Human Wound Technology and Sealed Sputum Suction" was retracted in 2023. Reasons: unreliable results or conclusions; concerns about the data; concerns about the peer review; concerns about the citations.

# Development of Training Videos Based on Virtual Reality Side-Cut High-Simulation Simulator of Human Wound Technology and Sealed Sputum Suction

**DOI:** 10.1155/2021/9985041

**Published:** 2021-09-08

**Authors:** Min Wang, Rong Rong, Ke Jia, Jing Li, Zhuohui Zhou, Wenxin Ge, Qing Zhang

**Affiliations:** ^1^Surgical, The Central Hospital of Wuhan, Wuhan 430014, Hubei, China; ^2^Orthopedic, The Central Hospital of Wuhan, Wuhan 430014, Hubei, China; ^3^Thoracic Surgery, The Central Hospital of Wuhan, Wuhan 430014, Hubei, China; ^4^Neurosurgery, The Central Hospital of Wuhan, Wuhan 430014, Hubei, China; ^5^Thoracic Surgery, The Central Hospital of Wuhan, Wuhan 430014, Hubei, China

## Abstract

The development of information technology and the advancement of the process of educational informatization have provided technical support for education and education reform. The virtual simulation teaching mode is no longer a new thing for people, and it is more and more accepted by people familiar with it. Induction and analysis of short message texts generated by students' online learning can fully understand students, make effective adjustments to the classroom, guide teachers' teaching practice, and optimize the classroom, thereby improving students' learning ability, practical ability, innovation ability, and collaboration. To study the effect of virtual simulation education on improving the skills of medical students, this paper is based on video training and education of virtual reality side-cut high-simulation simulator using case analysis and literature analysis methods. It collects data from databases and builds on online education. The model was developed, and a large number of relevant pieces of literature were read and analyzed through the literature survey method. The research results show that virtual simulation teaching can effectively improve students' technical thinking and ability. Students' technical thinking and ability are about 30% higher than traditional teaching methods, and the cooperation consciousness between students reaches 0.8 consciousness, which can solve the contradiction between popularization and improvement. And to solve the problems of polarization and transformation of underachievers, students' personalities can be fully displayed and developed, and education and teaching will be on the track of quality education. This shows that training videos based on virtual reality technology can play a very good role in improving students' technical mastery.

## 1. Introduction

With the rapid development of my country's economy and the continuous improvement of people's living standards, people's demand for medical technology is increasing and the complexity of surgery is becoming more and more complex. Low-level doctors are not competent without proper training [1]. According to the statistics of the Red Cross Society of our country, the number of deaths caused by medical injury accidents in China is about 400,000 each year, which is four times the number of deaths caused by traffic accidents. In particular, such delicate, complex, and difficult surgical operations as neurosurgery are easy to directly or indirectly cause varying degrees of harm to the patient. At present, the surgical skills of most surgeons are gradually mastered in the operating room by continuously performing actual surgical operations on real patients [2]. This traditional apprenticeship model of “pass, support, and bring-in” takes about 5–7 years to train surgeons with strong surgical and qualified skills. Obviously, such a training cycle cannot meet the needs of modern medical surgeons.

The article "Development of Training Videos Based on Virtual Reality Side-Cut High-Simulation Simulator of Human Wound Technology and Sealed Sputum Suction" was retracted in 2023. Reasons: unreliable results or conclusions; concerns about the data; concerns about the peer review; concerns about the citations.

The virtual surgery simulation system developed on the virtual reality technology has opened up a whole new field for solving the surgical skills training of junior doctors. Different from the traditional training methods of doctors, the virtual surgery simulation system is a new type of virtual reality application system that specializes in “distortion-free” simulation of various phenomena that may occur during surgery [3]. This type of surgical simulation system, with the help of a computer, provides trained physicians with three-dimensional anatomical and biomechanical properties that can be manipulated repeatedly without being restricted by time and space. We can provide various virtual “test materials.” This will greatly improve surgery. The efficiency of training and cost reduction provide new directions and ways to solve the problem of surgical training for medical students, interns, or junior doctors. With the continuous improvement of people's understanding of virtual surgery simulation systems, it has also been widely used in surgical navigation, surgical assistance, postoperative recovery training, and training videos [4].

In recent years, researchers have developed targeted virtual systems that can be used to simulate different operations based on the characteristics of different types of surgery. For example, Stanford University developed the virtual surgery simulation system for small blood vessels (usually 1 mm) and nerve sutures under the microscope, the Boston Surgical Planning Laboratory in the United States developed a virtual simulation system for simulating inner ear endoscopy, and the Canadian National Research Council developed the successful brain surgery virtual surgery simulation system, the Karlsruhe Laboratory in Germany developed a virtual minimally invasive surgery simulation training system using commercial simulation software, and the Swiss Tuchschmid et al. successfully developed a virtual hysteroscopy system after six years [5, 6]. At the same time, in order to further enhance the immersion and realism of the system, some scholars have introduced technologies such as augmented reality, boundary element, and automatic waves into the virtual surgery simulation system. Domestic virtual surgery started relatively late, and Xiong Yueshan and others developed a knee arthroscopic surgery simulation training system. The key problems of virtual surgery simulation such as geometric modeling, deformation calculation, and collision detection were studied deeply, and an improved spring particle model was proposed. It solves the phenomenon of “superelasticity” when the spring bears a large external force and has a good deformation visual effect. At the same time, the simulation of bleeding is added to the model, which further enhances the fidelity of the system [7]. On the one hand, these studies have enriched our understanding of college sports, but on the other hand, the conclusions of the experiment are not completely reasonable. The research samples are small and the conclusions are not universal enough to be convincing.

The article "Development of Training Videos Based on Virtual Reality Side-Cut High-Simulation Simulator of Human Wound Technology and Sealed Sputum Suction" was retracted in 2023. Reasons: unreliable results or conclusions; concerns about the data; concerns about the peer review; concerns about the citations.

The innovation of this paper is that, in order to further enhance the immersion and interactivity of the virtual surgery simulation system, this paper designs a general virtual surgery simulation platform. The platform is designed according to the physiological structure of the human body, allowing users to be completely immersed in the virtual operation process, free from external light, sound, and other uncontrollable factors. A surface cutting method based on boundary splitting is proposed. The difficulty of realizing surface patch splitting based on edge splitting points is to record the cutting state and maintain the consistency of the vertex state in the physical model. The cutting trajectory can be well described by recording the position and sequence of the boundary split points. This is the basis for the later insertion of internal vertices and the generation of new surfaces, as well as the basis for the topological reconstruction of internal point sets.

## 2. Training Video Development Method

### 2.1. Virtual Reality Side-Cut High-Simulation Simulator of Human Wound Technology

Virtual reality technology is an interactive dynamic virtual environment built by sensor technology, computers, and artificial intelligence that acts on human perception to make people feel like they are there. Virtual practice is the product of the rapid development of computer, Internet, information technology, and virtual reality technology. This type of practice is separated from scientific practice and forms a new practice mode [8]. The usual virtual practice refers to the purposeful and two-way object-oriented perceptual activities of the subject in the virtual environment through digital media. Different from traditional practice, the virtual practice has the characteristics of real-time interaction, virtual reality, and communication immersion. Its practice process is not restricted by external objective conditions, transcends the limitations of time and space, and can act on objective reality [9].

The article "Development of Training Videos Based on Virtual Reality Side-Cut High-Simulation Simulator of Human Wound Technology and Sealed Sputum Suction" was retracted in 2023. Reasons: unreliable results or conclusions; concerns about the data; concerns about the peer review; concerns about the citations.

Compared with traditional surgeon training methods, virtual surgery simulation systems developed on the basis of virtual reality have the advantages of low cost, high efficiency, repeatable exercises, and freedom from time and space and ethical constraints and are becoming a research hotspot in the medical field and cutting-edge topics [10]. The virtual surgery simulation system uses computer technology to create realistic surgical scenes in the same virtual environment as in the real world. This allows users to interact with virtual tissues and organs through force feedback devices to complete operations such as palpation, cutting, and tearing and suction training, so as to quickly and effectively improve the surgical skills of interns, new doctors, and other junior doctors. At the same time, it can also be used as an auxiliary means to optimize the surgical plan and perform intraoperative navigation. Virtual surgery simulation is the expansion and extension of virtual reality technology in the medical field, opening up a new field for doctor training, surgical navigation, and telemedicine. The high-simulation simulator in this paper is mainly prepared through the following steps [11].

The establishment of a three-dimensional hybrid model: the high-simulation human simulator model used in this paper is a hybrid model that combines surface models with mesh-free technology. This model not only maintains the surface triangular mesh used to represent the contour information of the object but also records the point set used to describe the internal structure of the object [12]. In the process of constructing the hybrid model, an adaptive meshing method is used to automatically calculate the point set representing the internal structure.

Collision detection and response: the collision detection part uses the simplest and fastest bounding box method, but proposing a hypothesis of spatiotemporal consistency improves the efficiency of the original algorithm, and the reliability of this hypothesis in real applications is experimental.

The article "Development of Training Videos Based on Virtual Reality Side-Cut High-Simulation Simulator of Human Wound Technology and Sealed Sputum Suction" was retracted in 2023. Reasons: unreliable results or conclusions; concerns about the data; concerns about the peer review; concerns about the citations.

Establishment of deformation model: a mass point-spring model is established on the current hybrid grid structure, and a restoring force based on the relative position of the mass points is added to maintain the volume of the model. Experiments have proved that the spring model based on the current hybrid model structure is more robust than the regular grid structure.

Grid splitting and reconstruction: the splitting of the mesh during the cutting process includes the splitting of the triangles on the surface and the generation of new internal vertices. The two data structures maintained by the current hybrid model during cutting need to be updated simultaneously [13]. In the process of surface splitting, the outer patch adopts a splitting method based on the boundary splitting point, while the inner surface adaptively generates new vertices and meshes by tracking the cutting surface of the virtual instrument. To ensure the quality of the mesh after cutting, the vertices are moved during the segmentation and vertex insertion process to improve the quality of the reconstructed mesh.

Speed up the learning progress of surgeons and prevent the potential danger of internship or low-age surgeons that can easily cause harm to patients. For intern or low-age surgical surgeons, due to various objective factors, they have very few opportunities for actual surgical training (some doctors have very limited surgical experience even if they have some surgical experience) and lack actual surgical experience. It is difficult to quickly improve surgical skills in a short time [14]. The virtual surgery simulation system allows doctors to perform unlimited training in a virtual environment, significantly improving their surgical capabilities. Moreover, the training object is a fictitious illusion, which will not cause any substantial harm to the patient.

### 2.2. Sealed Sputum Suction

Another important measure in respiratory management is endotracheal sputum suction, the main purpose of which is to suck out secretions in the airway in time to maintain unobstructed airway. Therefore, intratracheal sputum aspiration is very important for maintaining ventilatory function and preventing and treating lung infections. Sputum suction in the airway includes two types: open suction and closed suction. The traditional suction method is an open suction method, which uses a disposable suction tube. During clinical use, people find that this method requires the interruption of the ventilator treatment and also brings problems such as cross-infection and environmental pollution [15].

Closed suction requires the help of a sterile auxiliary device. Compared with open suction, closed suction has the following advantages:

1. Open sputum suction requires disconnection of the ventilator or oxygen inhalation device, which may cause a large decrease in lung capacity, alveolar collapse, decreased arterial oxygen saturation, increased reflex heart rate, increased blood pressure, and so on for high-risk adverse reactions. In patients with hypoxic saturation, the use of an open suction system is likely to cause lung collapse; closed suction can maintain the continuity of mechanical ventilation and oxygenation during the suction process, with minimal impact on the patient's lung capacity and no significant decrease in SpO_2_, to avoid patients with hypoxia and CO_2_ retention. For neurosurgery patients, it can also prevent cerebral vasoconstriction, decrease in cerebral blood flow, decrease in cerebral perfusion pressure, and increase in intracranial pressure [16].
2. The closed suction tube has a protective cover that prevents direct contact with the suction tube during suction, reducing the risk of contamination and not increasing the risk of ventilator-related pneumonia.
3. There is no need for routine daily replacement. Compared with the disposable suction tube, there is no need to check the suction tube, wear sterile gloves, and do other steps. According to related research reports, the time of closed suction is longer than that of open suction (shortened by about 1 minute). This is a very important guarantee that hypoxic-sensitive patients (such as brainstem hemorrhage, brainstem tumors, and other patients with respiratory center effects) maintain oxygenation and ensure a continuous oxygen supply. It also saves time. And human power improves the work efficiency of nurses [17].
4. During open sputum suction, the airway communicates with the outside air, and the sputum splashes, causing pollution to the hands, clothes, objects, and the environment of the medical staff. If the sterilization and isolation are not in place, the medical staff's aseptic technique is not rigorous, which can increase the lungs. Due to the application of the protective cover, the closed sputum suction reduces the chance of medical staff contacting infectious secretions, effectively avoids cross-infection, prevents the occurrence of nosocomial infections, and improves the safety of medical care.

The article "Development of Training Videos Based on Virtual Reality Side-Cut High-Simulation Simulator of Human Wound Technology and Sealed Sputum Suction" was retracted in 2023. Reasons: unreliable results or conclusions; concerns about the data; concerns about the peer review; concerns about the citations.

Airway management technology mainly involves artificial airway fixation, secretion removal, balloon management, airway humidification, and so on. Among them, adequate humidification and necessary sputum suction are important measures for the management of artificial airway patients' secretions. At present, the humidification device and sputum suction method have undergone revolutionary development with the upgrading of science and technology, and there are also certain controversies. The traditional airway humidification and sputum suction methods are artificial nose and open endotracheal sputum suction. Currently, they are commonly used in clinical practice, but they also have many drawbacks that can increase the risk of airways in patients such as pneumonia. The heated humidifier with a heated guidewire system can reach 37°C and the humidity between 42 mg/L and 44 mg/L. It meets the requirements of relevant documents and guidelines. It is an outstanding representative of modern constant temperature humidification systems [18]. The closed suction method has more advantages than the open suction method in terms of ease of operation, prevention of infection, and maintenance of blood oxygen saturation. In this study, the combined use of a heated humidifier and a closed sputum suction method was compared with the traditional artificial nose combined with an open sputum suction method. The research was comprehensively considered from the patient's sputum viscosity, moisturizing effect, sputum, incidence of lung infection, artificial airway indwelling time, NSICU hospitalization time, and other indicators [19].

The closed suction method avoids the problem of lung collapse caused by the open suction system in patients with high-risk hypoxic saturation and reduces the risk of contamination. Adequate moisturization and effective sputum suction are beneficial to reduce sputum, pulmonary infection, and so on and provide a good moisturizing effect, thereby promoting patient recovery, shortening the length of hospitalization, and reducing hospitalization costs [20].

### 2.3. Simulation Model Establishment

From the nature of the human tissue model, a complete human tissue model is composed of two parts: a geometric model and a physical model. The so-called geometric model refers to a model used to describe geometric information such as the shape, size, position, and structure of an object. The physical model adds corresponding physical properties to the basis of the geometric model, such as the mass and density of the object [21]. Therefore, in order to establish a human tissue model, the geometric model of the human tissue must be reconstructed first. With the rapid development of large-scale medical imaging equipment and the improvement of three-dimensional object shape detection technology, the three-dimensional geometric modeling of human soft tissue has become an important subject in the field of modern graphics and imaging, which has attracted extensive attention and in-depth research [22]. The reconstruction technology of the 3D geometric model of human tissue is to study how to obtain 3D information of soft tissue shape and position in space through the two-dimensional medical image information of human soft tissue and finally obtain the spatial 3D model of soft tissue [23]. Contrary to the general model building process, the three-dimensional reconstruction of soft tissue is to map the existing real human soft tissue to the three-dimensional geometric model in the computer to construct the three-dimensional virtual model of the computer, which is called reverse engineering or reverse technology. The equation is transformed into the following formula:

(1) $$\begin{array}{c} R=b_{o}^{2}\left[1+\frac{w^{\prime \prime }}{w^{\prime }}\frac{au}{a\;d}+\cdots \right]\frac{a^{2}r}{ad^{2}}. \end{array}$$

Among them, *R* particle represents the influence on time *t*; *d* is the distance; and *b*02 is the speed. The relevant equation is

(2) $$\begin{array}{c} \eta_{2}=-\frac{w^{\prime \prime }}{2w^{\prime }}. \end{array}$$

Variants of nonlinear equations of motion are

(3) $$\begin{array}{c} \sum_{n=1}^{i}\left(\vartheta r_{n}*w_{n}r_{n}+\vartheta \mu_{n}j_{n}\mu_{n}\right)-\sum_{j=1}^{i}\vartheta \theta_{n}\nu_{n}-\vartheta r_{i}*S_{i}=Q. \end{array}$$

The solution of the equation is

(4) $$\begin{array}{c} R=R_{1}\cos\left(qx-wd\right)-\frac{1}{4}\eta_{2}q^{2}R_{2}x\;\sin\;2\left(qx-wd\right)+\cdots . \end{array}$$

The relationship between *R*_2_ and *R*_3_ can be obtained as follows:

(5) $$\begin{array}{c} R_{2}=\left(\frac{\eta_{2}}{4}\right)d^{2}R_{1}^{2}x,\\ dm=\frac{g_{m}{\left(\varpi /\Omega \right)}^{2}}{\sqrt{\left[1-{\left(\varpi /\Omega \right)}^{2}+{\left(2\phi \varpi /\Omega \right)}^{2}\right]}}. \end{array}$$

Calculation is as follows:

(6) $$\begin{array}{c} \delta_{i}=st\;\cos\left[\frac{\sum_{j=1}^{3}\left(x_{i,j}*x_{j,0}\right)}{{\left(\sum_{j=1}^{3}x_{i,j}^{2}\right)}^{1/2}*{\left(\sum_{x_{j,0}^{2}}^{3}x_{j,0}^{2}\right)}^{1/2}}\right], \end{array}$$

where *a* represents the weight and the range is between [0, 1]. The calculation is as follows:

(7) $$\begin{array}{c} F=\frac{\sum \left(q_{rp,rpn}-q_{rpm}\right)\left(q_{uq,uqn}-q_{uq}\right)}{\sum_{n=1}^{n}{\left(q_{r}-q_{uq}\right)}^{2}\sqrt{\sum {\left(q_{uq,uqm}-q_{uq}\right)}^{2}}}. \end{array}$$

Using image segmentation methods, users can select specific areas of interest or target organs from medical image data and calculate segmentation results in an accurate 3D model [24]. It is necessary to adjust the spring model's various force parameters to control the spring's return characteristics and stability and shorten the time step in the simulation as much as possible to reduce the simulation error in the discretization process

(8) $$\begin{array}{c} \alpha \left(z\right)=1+\alpha_{1}z^{-1}+\alpha_{2}z^{-2}+\cdots +\alpha_{n}z^{-n},\\ \beta_{ij}\left(z\right)=\beta_{ij}^{0}+\beta_{ij}^{1}z^{-1}+\beta_{ij}^{2}z^{-2}+\cdots +\beta_{ij}^{n}z^{-n}. \end{array}$$

Its optimal value is

(9) $$\begin{array}{c} ZM\left(\vartheta \right)Z^{Z}\vartheta -Zc\left(\vartheta ,\dot{\vartheta }\right)=\delta +ZB\left(\vartheta \right)F_{n}. \end{array}$$

The material parameters are

(10) $$\begin{array}{c} y\left(kT+t_{i}\right)=\frac{1}{\alpha \left(z\right)}\sum_{j=1}^{r}\beta_{ij}\left(z\right)\bar{u}\left(kT+t_{j-1}\right)+v\left(kT+t_{i}\right). \end{array}$$

Voxelization is a necessary pretreatment process for volume graphics. Its purpose is to convert the continuous geometric shape of an object into a voxel representation that is closer to the object [25]. This voxel representation method not only contains the surface information of the model but also describes the internal properties of the object (such as density and quality). It can be considered as an extension of two-dimensional pixels in three-dimensional space.

The article "Development of Training Videos Based on Virtual Reality Side-Cut High-Simulation Simulator of Human Wound Technology and Sealed Sputum Suction" was retracted in 2023. Reasons: unreliable results or conclusions; concerns about the data; concerns about the peer review; concerns about the citations.

## 3. Training Video Teaching Experiment

### 3.1. The Purpose of the Experiment

This paper makes full use of the research results in the field of virtual reality technology to achieve the development of sealed sputum suction training videos. Through in-depth research on memory problems in medical education, an optimized sealed sputum suction training system is constructed, and the technology of high-simulation human wounds based on virtual reality lateral cutting is promoted, and the feasibility and scientific opinions are further put forward. By comparing the training effects of different methods for medical students in the city's universities, it helps the current medical system to build a better training system.

### 3.2. Virtual Model Construction

For virtual surgery simulation systems, the reconstruction of a very detailed 3D soft tissue model is the most immediate and effective way to improve the user's visual presence. The modeling process is mainly divided into two stages: the first step is to construct a three-dimensional surface geometric model of human soft tissue based on two-dimensional CT images; this step transforms from two-dimensional grayscale images into three-dimensional models. The second step is to use morphing continuous deformation technology to titrate the 3D surface model from the 3D surface soft geometric model of human soft tissue to obtain the human soft tissue model containing the internal point cloud.

### 3.3. Model Voxelization

Volume representation uses 3D volume units to describe the entire object, which is similar to the pixels of a 2D digital image. Voxelization is a necessary pretreatment process for volume graphics. Its purpose is to convert the continuous geometric shape of an object into a voxel representation that is closer to the object. This voxel representation method not only contains the surface information of the model but also describes the internal properties of the object (such as density and quality). It can be considered as an extension of two-dimensional pixels in three-dimensional space.

The article "Development of Training Videos Based on Virtual Reality Side-Cut High-Simulation Simulator of Human Wound Technology and Sealed Sputum Suction" was retracted in 2023. Reasons: unreliable results or conclusions; concerns about the data; concerns about the peer review; concerns about the citations.

### 3.4. Comprehensive Evaluation Model

At present, there are two main evaluation models: one is the main factor highlight model, and the other is the weighted average model. If the weight of a single factor is significant and there are dominant factors in the evaluation factors, you can choose the prominent main factor model; if the weight of the evaluation factors is relatively average, you can choose the weighted average model. These two models have their own characteristics. In the specific implementation process, the two methods can be implemented separately. We selected evaluators with more than 2 years of evaluation experience to participate and compared the results of the two models.

## 4. Analysis of Teaching and Training Experiments

### 4.1. Changes in Training and Teaching

As time changes, people have made many attempts on teaching and training methods. Through questionnaire surveys and consulting a large number of materials, we have collected statistics on the most commonly used teaching and training methods in recent years and transformed them into specific methods through model calculations. Values and data are shown in Table 1.

From Figure 1, we can see that, in the teaching and training methods, the groups used in various methods are basically similar, and there is no uniformity of these types of methods. As time changes, the groups of people using different methods are also constantly changing. Among them, the method based on the information processing teaching model used in this article shows a trend of first decline and then rise, from 2.3 in 2014 to 2.66 in 2019, and 2015 was the largest number of people using this method. We show the different growth trends from 2014 to 2019, as shown in Table 2.

From Figure 2, we can see that the various teaching and training methods used in the past five years have relatively large changes, but the virtual reality technology-based simulation human teaching method used in this paper has appeared in the past five years. It is an upward trend. Among them, the largest increase was in 2018, with a range of 0.16, which also shows that teaching methods based on virtual reality technology are becoming more and more accepted by people.

The article "Development of Training Videos Based on Virtual Reality Side-Cut High-Simulation Simulator of Human Wound Technology and Sealed Sputum Suction" was retracted in 2023. Reasons: unreliable results or conclusions; concerns about the data; concerns about the peer review; concerns about the citations.

### 4.2. Highly Simulated Human Wound Technology

This paper adopts the high-simulation human simulating wound technology based on virtual technology. By distinguishing the artificial humans of different simulation forms and comparing the wound parameters under different simulation levels, it can be clearly seen that each of the high-simulation humans is different. All simulation parameters are higher than the others. The group classification parameters are shown in Table 3.

As shown in Table 3, we divide the simulated humans into three groups through dynamic capture and static capture parameters and compare them with the parameters of the actual human body. From the table, we can clearly see that there are obvious differences in the parameters of different types of patients. Inferior simulated human data are very different from real humans, while the data parameters of high simulated humans are basically close to real humans, which can simulate the effect of the human body. We analyze the incisions of high-simulation people, as shown in Figures 3 and 4.

From the renderings in Figures 4 and 5, we can see that, by simulating the incision of a high-simulation human, the incision and the rendered image are basically close to the real effect. Although there are still some gaps, the error is within the allowable range. And for training and teaching, it can improve students' familiarity with the human body and increase their interest in learning.

### 4.3. Teaching and Training

We divide these students into six classes, divide these six classes into three groups, and carry out a three-month teaching training according to different teaching methods. After the teaching is over, statistics of the students' relevant data are carried out. The postdata are shown in Table 4.

From Figure 5, we can see that, after the teaching, the male students' mastery of artistic skills has improved to a certain extent. The effect of online teaching is far better than offline teaching. Art teaching based on the Internet and virtual simulation technology achieves the best effect, which is twice as high as before teaching and more than 50% higher than other teaching methods. In order to verify the correctness of the results, we also conducted statistics on the teaching data of female students, as shown in Table 5.

From Figure 6, we can confirm again that, after teaching, students' mastery of training skills has an excellent improvement effect, and the effect of teaching based on virtual simulation technology is better than that of the other two teaching methods. Male students have improved more than female students in some aspects, but overall, female students' overall improvement after teaching is slightly greater than that of male students.

The article "Development of Training Videos Based on Virtual Reality Side-Cut High-Simulation Simulator of Human Wound Technology and Sealed Sputum Suction" was retracted in 2023. Reasons: unreliable results or conclusions; concerns about the data; concerns about the peer review; concerns about the citations.

### 4.4. Survey of Teaching Views

We have made statistics on the views of the students and teachers of these classes on the virtual simulation teaching mode and understood their views on these teachings. The statistics are shown in Table 6.

From the table, we can see that, in the Internet-based simulation teaching, the satisfaction of students and teachers is relatively high, and the total proportion of dissatisfied students and teaching is about 10%. For the convenience of comparison, we have also made statistics on the satisfaction of traditional teaching, as shown in Table 7.

From Figure 7, we can see that the satisfaction of traditional teaching is not high, which is much lower than that of simulation teaching. Simulation teaching is a kind of teaching. According to the development of main media and information technology, multimedia network teaching belongs to the third generation of distance teaching. Simulated online teaching is the product of the development of modern computer network technology and multimedia technology to a certain extent, and it is extremely attractive to students.

## 5. Conclusion

Based on the study of the deformation characteristics and force feedback characteristics of the soft anthropomorphic wound technology in the actual operation, the soft tissue cutting model is established by the meshless method, and the complete process of the cutting is realistically simulated and reproduced by making a video. Of course, this paper also has some shortcomings. The texture of the 3D soft tissue model reconstructed in this paper is relatively simple and not detailed enough, and it cannot fully and accurately simulate the real anatomical structure and physiological function of the tissue. The distribution and direction of blood vessels and ducts in the tissues cannot be shown in the model. When the complexity of the cutting model is further increased, for example, after models such as bleeding and hemostasis are added, it is difficult to meet the real-time requirements of the system by simple serial calculation.

## Figures and Tables

**Figure 1:** Changes in teaching and training methods.

**Figure 2:** Growth trend of mining methods.

**Figure 3:** Artificial human incision (from Baidu: image.baidu.com).

**Figure 4:** Discrete effect of artificial human incision. (a) Discrete postrendering effect. (b) Cut rendering effect 1. (c) Cut rendering effect 2 (from Baidu: image.baidu.com).

**Figure 5:** Changes of male students after teaching.

**Figure 6:** Female students after teaching.

The article "Development of Training Videos Based on Virtual Reality Side-Cut High-Simulation Simulator of Human Wound Technology and Sealed Sputum Suction" was retracted in 2023. Reasons: unreliable results or conclusions; concerns about the data; concerns about the peer review; concerns about the citations.

**Figure 7:** Traditional teaching satisfaction survey.

**Table 1:** Vulnerability mining method.

	2012	2013	2014	2015	2016	2017	2018	2019	2020
Information processing	1.94	2.38	2.13	2.21	2.29	2.34	1.97	2.06	2.2
Personality development	2.35	1.8	2.46	1.97	2.36	2.03	1.94	2.2	1.96
Social interaction	1.99	2.08	1.98	1.89	2.09	2.49	1.8	2.19	1.94
Behavior modification	2.15	2.45	2.25	2.1	2.24	2.2	2.15	2.46	1.81
Online teaching	1.93	2.35	1.97	2.45	2.28	2.37	2.17	2.08	1.92
Traditional teaching	2	2.26	2.33	2.3	1.86	2.35	1.95	2.08	2.12
Virtual reality	2.36	2.13	2.27	2.3	2.42	2.46	2.47	2.63	2.66

**Table 2:** Changes in different methods.

	2015	2016	2017	2018	2019
Information processing	0.08	0.05	−0.37	0.09	0.06
Personality development	0.39	−0.33	−0.09	0.18	−0.26
Social interaction	0.2	0.4	−0.69	0.39	−0.25
Behavior modification	0.13	−0.04	−0.05	0.31	−0.65
Online teaching	−0.27	0.09	−0.2	−0.09	−0.16
Traditional teaching	−0.44	0.49	−0.4	0.13	0.04

**Table 3:** Patient SPN classification.

	Low emulation	General simulation	High-simulation person	Entity data	*P*
Optic nerve	73.88 ± 3.77	78.56 ± 8.23	88.35 ± 5.78	89.26 ± 2.38	*P* < 0.05
Filter	5.69 ± 4.32	8.79 ± 3.58	17.23 ± 4.85	15.32 ± 3.51	*P* < 0.05
Daily life	12.34 ± 5.81	7.56 ± 4.25	8.48 ± 3.45	5.23 ± 2.01	*P* < 0.05
Motion capture	9.24 ± 3.52	13.52 ± 4.72	27.89 ± 5.32	25.34 ± 3.17	*P* < 0.05
Static capture	4.25 ± 2.35	9.25 ± 3.14	12.47 ± 4.91	11.37 ± 4.17	*P* < 0.05

**Table 4:** Male students after teaching.

Teaching methods	Class	Creative thinking	Learning attitude	Learning ability	Basic ability	Painting	Cultural lessons
Offline teaching	Class 1	2.35	2.01	1.86	2.15	2.29	2.11
	Class 2	1.87	2	2.04	1.89	2.11	2.36

General online teaching	Class 3	3.6	3.82	3.43	3.32	3.37	3.42
	Class 4	3.81	4.07	4.01	4.01	4.16	3.78

Virtual simulation teaching	Class 5	4.84	5	4.77	4.88	4.87	5.35
	Class 6	5.6	5.63	5.84	5.37	5.13	5.26

**Table 5:** Changes of female students after teaching.

Teaching methods	Class	Creative thinking	Learning attitude	Learning ability	Basic ability	Painting	Cultural lessons
Offline teaching	Class 1	3.08	3.16	2.86	2.73	2.81	3.39
	Class 2	3.8	3.81	3.84	3.57	3.89	3.24

General online teaching	Class 3	4.82	4.42	4.41	4.94	4.91	4.24
	Class 4	4.89	5.17	4.7	4.91	4.78	4.98

Virtual simulation online teaching	Class 5	6.14	6.22	5.7	6.13	5.77	5.89
	Class 6	6.55	6.82	6.62	6.3	6.85	6.42

**Table 6:** Attitudes towards multimedia teaching.

	Very dissatisfied	Not satisfied	General	Okay	Satisfaction	Very satisfied
Class 1	2	4	12	14	17	19
Class 2	2	3	7	12	21	20
Class 3	3	5	13	12	20	24
Class 4	5	5	12	17	19	20
Class 5	1	6	8	11	22	21
Class 6	2	2	13	11	17	19

**Table 7:** Traditional teaching satisfaction.

	Very dissatisfied	Not satisfied	General	Okay	Satisfaction	Very satisfied
Class 1	6	5	22	14	6	7
Class 2	7	2	19	11	7	5
Class 3	9	7	25	15	9	10
Class 4	7	3	12	19	10	9
Class 5	4	6	18	19	11	7
Class 6	7	4	20	21	8	12

The article "Development of Training Videos Based on Virtual Reality Side-Cut High-Simulation Simulator of Human Wound Technology and Sealed Sputum Suction" was retracted in 2023. Reasons: unreliable results or conclusions; concerns about the data; concerns about the peer review; concerns about the citations.

## Data Availability

No data were used to support this study.
